This article has been retracted.

# The long noncoding RNA AK002107 negatively modulates miR‐140‐5p and targets TGFBR1 to induce epithelial–mesenchymal transition in hepatocellular carcinoma

**DOI:** 10.1002/1878-0261.12487

**Published:** 2019-04-11

**Authors:** Yun‐Hua Tang, Guo‐Lin He, Shan‐Zhou Huang, Ke‐Bo Zhong, Hui Liao, Lei Cai, Yi Gao, Zhen‐Wei Peng, Shun‐Jun Fu

**Affiliations:** ^1^ Organ Transplant Center the First Affiliated Hospital Sun Yat‐sen University Guangzhou China; ^2^ Department of Hepatobiliary Surgery II Zhujiang Hospital Southern Medical University Guangzhou China; ^3^ Department of Oncology the First Affiliated Hospital Sun Yat‐sen University Guangzhou China

**Keywords:** epithelial–mesenchymal transition, hepatocellular carcinoma, lncRNA AK002107, miR‐140‐5p

## Abstract

The abnormal expression of long noncoding RNAs (lncRNAs) is associated with human carcinoma. The present study aimed to investigate the mechanisms underlying the function of lncRNA AK002107 in the progression of hepatocellular carcinoma (HCC). The differential expression of lncRNAs between HCC and paired nontumor tissues was identified using microarrays, and the correlation between the expression of lncRNA AK002107 and the clinical prognosis of HCC was analyzed. We investigated the role of lncRNA AK002107 in HCC tumor biology *in vitro* using 3‐(4,5‐dimethylthiazol‐2‐yl)‐2,5‐diphenyl‐tetrazolium bromide (MTT), colony formation, and Matrigel invasion assays and *in vivo* by assessing the growth of xenografted HCC tumors. The potential microRNAs that interact with lncRNA AK002107 were identified using online tools and were verified using PCR and luciferase reporter assay. The levels of TGFBR1, E‐cadherin, and vimentin were determined using western blot assays. We then further investigated the correlation between expression of lncRNA AK002107 with miR‐140‐5p and TGFBR1 expression in HCC tissues. The expression of lncRNA AK002107 is frequently upregulated in HCC samples and cell lines. Patients with HCC who have elevated lncRNA AK002107 expression exhibit poorer overall survival and disease‐free survival. Silencing lncRNA AK002107 expression significantly inhibited HCC cell proliferation, colony formation, and invasion both *in vitro* and *in vivo*. Furthermore, lncRNA AK002107 directly binds to miR‐140‐5p and significantly inhibits miR‐140‐5p expression. The functions of lncRNA AK002107 in cell growth and tumor invasion are mediated via miR‐140‐5p. lncRNA AK002107 upregulated TGFBR1 expression and then induced epithelial–mesenchymal transition (EMT) by inhibiting miR‐140‐5p expression. The expression of lncRNA AK002107 inversely correlated with miR‐140‐5p expression and positively correlated with TGFBR1 expression in HCC tissues. In summary, lncRNA AK002107 functions as an oncogene in tumors by inhibiting miR‐140‐5p, targeting TGFBR1, and then inducing EMT. The lncRNA AK002107/miR‐140‐5p/TGFBR1/EMT regulatory network may be a valuable target for the development of novel diagnostic and treatment methods for HCC.

**Abbreviations**
EMT: epithelial–mesenchymal transition
HCC: hepatocellular carcinoma
lncRNAs: long noncoding RNAs
miRNAs: microRNAs

## 1 Introduction

Hepatocellular carcinoma (HCC) is one of the most common gastrointestinal cancers worldwide (Maluccio and Covey, 2012). Approximately 55% of all patients with HCC worldwide reside in China (Yuen *et al*., 2009). Although hepatic resection and liver transplantation are effective and radical treatments for patients with HCC, a large proportion of patients have a poor 5‐year survival rate and a high recurrence rate due to a high rate of intrahepatic and extrahepatic metastases (Budhu *et al*., 2006). Therefore, the identification of novel prognostic molecular markers is urgently needed to establish new therapeutic targets for successful treatment strategies and to gain a greater understanding of the molecular mechanisms of hepatocarcinogenesis.

Long noncoding RNAs (lncRNAs) constitute a class of non‐protein‐coding transcripts with a length greater than 200 nucleotides (Tay *et al*., 2014). Based on accumulating evidence, dysregulated lncRNA expression is frequently observed in many diseases and is involved in multiple biological processes, such as cellular proliferation, apoptosis, and migration (Mercer *et al*., 2009). Recently, lncRNA expression profiling has shown great potential in determining the diagnosis and prognosis of human carcinomas, such as colon cancer (Takahashi *et al*., 2014), breast cancer (Huang *et al*., 2014), and HCC (Yuan *et al*., 2012), and lncRNAs may serve as effective therapeutic targets for interventions. Although thousands of lncRNAs have been identified, the functions of most lncRNAs remain unknown.

In the current study, the differences in lncRNA expression profiles between HCC tissues and tumor‐adjacent nontumor tissues were assessed, and the potential relationships between lncRNA expression levels and the clinicopathological characteristics of patients with HCC were investigated. Moreover, silencing lncRNA AK002107 inhibited HCC cell proliferation, colony formation, and invasion. Furthermore, lncRNA AK002107 was found to play a functional role in epithelial–mesenchymal transition (EMT) induction by inhibiting miR‐140‐5p expression and then upregulating TGFBR1 expression. These results provide new insights into the roles of lncRNAs in the development of HCC and highlight the potential application of lncRNA AK002107 in the treatment of HCC.

## 2 Materials and methods

### 2.1 Tissue specimens

Two independent cohorts of 135 patients with HCC were enrolled in our study. In cohort 1, 35 fresh HCC samples and adjacent noncancerous tissues were collected from 35 patients who initially underwent liver resection at the First Affiliated Hospital of Sun Yat‐sen University (Guangzhou, China) between May 2012 and August 2012; five HBV‐related HCC tissues and corresponding noncancerous tissues were used for the microarray analysis (Table S1). Another 30 HCC tissues and corresponding noncancerous tissues were used for further validation and the correlation analysis (Table S2). In cohort 2, 100 HCC tissues from patients who underwent liver transplantation between January 2009 and July 2013 at the same hospital were used for the survival analysis. The study protocol followed the Ethical Guidelines of the Declaration of Helsinki. All patients gave written informed consent on the use of clinical specimens for medical research. This study was approved by the Ethics Committee of the First Affiliated Hospital of Sun Yat‐sen University. The patients’ clinical information is presented in Table 1.

**Table 1:** Relationship between the expression of lncRNA‐AK002107 and clinicopathological characteristics. AFP, alpha fetoprotein; HBsAg, Hepatitis B surface antigen. The categorical parameters were compared with the chi‐square test or Fisher's exact test and analysis of variance as appropriate

Category	Subcategory	Cases	lncRNA‐AK002107 expression		*P*‐value
			Low (*n* = 39)	High (*n* = 61)	
Gender	Male	94	35	59	0.152
	Female	6	4	2	
Age (years)	≤ 50	50	16	34	0.151
	< 50	50	23	27	
HBsAg	Positive	92	36	56	0.928
	Negative	8	3	5	
Child‐Pugh stage	A	63	25	38	< 0.001**
	B	32	10	22	
	C	5	4	1	
Preoperative tumor therapy	Yes	44	16	28	0.632
	No	56	23	33	
AFP (ng·mL^−1^)	≤ 400	60	31	29	0.001**
	> 400	40	8	32	
Size of largest tumor (cm)	≤ 5	52	28	24	< 0.001**
	5–8	19	4	15	
	> 8	29	7	22	
Tumor number	≤ 3	80	30	50	0.539
	> 3	20	9	11	
Edmonson grading	I–II	70	30	40	0.227
	III–IV	30	9	21	
Macrovascular invasion	Yes	25	1	24	< 0.001**
	No	75	38	37	
Microvascular invasion	Yes	19	3	16	
	No	81	35	46	0.027*

^*^ *P* < 0.05; ^**^ *P * 0.01.

### 2.2 Microarrays and computational analysis

Fresh samples from five HBV‐related HCC tissues and corresponding noncancerous tissues were randomly selected for the microarray analysis. Total RNA was extracted from the tissue specimens using TRIzol (Invitrogen, Carlsbad, CA, USA) and purified with the RNeasy Mini Kit (Qiagen p/n 74104, Hilden, Germany). Then, each sample was amplified and transcribed into fluorescent cRNAs along the entire length of the transcripts without a 3′ bias using a random priming method. The labeled cRNAs were hybridized onto the Human lncRNA Array v2.0 (8 × 60K, Arraystar). After washing the array, the slides were scanned with an Agilent Scanner G2505C (Agilent p/n G2505C, Santa Clara, CA, USA). The data were recorded using Agilent feature extraction software (version 11.0.1.1). Further data analyses were performed using Agilent genespring gx v11.5.1 software. A hierarchical clustering analysis was performed between the HCC samples and the corresponding noncancerous tissue samples to identify significantly differentially expressed lncRNAs.

### 2.3 *In situ* hybridization

*In situ* hybridization (ISH) was performed by employing an ISH kit from BersinBio (Guangzhou, China), as previously described (Hu *et al*., 2014). Samples were fixed with 4% paraformaldehyde (DEPC, Servicebio) for 2–12 h. Paraffin sections were generated to perform the hybridization reaction. The probe was designed, synthesized, and labeled with digoxin by BersinBio, and the probe sequence was 5′‐DigN‐GAACTGTAAAGTGCCTTTATAAC‐3′‐DigN. The 5′ and 3′ UTRs were labeled with digoxin. Then, sections were placed in boiling water for 15 min and cooled to room temperature. Specimens were incubated at 37 °C for 30 min with 20 μg·mL^−1^ Proteinase K and then rinsed three times with PBS. Prehybridization was conducted at 37 °C for 1 h in hybridization buffer. Then, the prehybridization buffer was replaced with fresh hybridization buffer containing 8 ng·mL^−1^ of the corresponding probe, and the specimens were incubated at 37 °C overnight. After washing, the specimens were incubated at room temperature in blocking buffer containing BSA for 30 min. Then, the specimens were incubated with an anti‐DIG/AP antibody (Jackson, Pennsylvania, PA, USA) at 37 °C for 40 min. The color reactions were conducted using BCIP/Nitro Blue tetrazolium (Boster, Wuhan, China). Specimens were stained with nuclear fast red (Servicebio) to visualize the cell nuclei. The stained specimens were mounted in Neutral Balsam (Sinopharm Chemical Reagent Co., Ltd., Shanghai, China) and examined under a bright‐field microscope. ISH staining was evaluated by two pathologists, and the standard used to score the staining intensity was 0 (negative), 1 (weak), 2 (medium), and 3 (strong). The scores for the extent of staining were 0 (0%), 1 (1–25%), 2 (26–50%), 3 (51–75%), and 4 (76–100%). The total scores reflect the intensity and extent scores and range from 0 to 7 points. We considered total scores of 3 or more than 3 points the high expression group.

### 2.4 Cell lines

The HepG2 human HCC cell line was purchased from the American Type Culture Collection (ATCC; Rockville, MD, USA). The MHCC97H, MHCC97L, SMMC7721, Hep3B, and BEL7402 human HCC cell lines and LO_2_ immortalized normal liver cell line were obtained from the Institute of Biochemistry and Cell Biology (Chinese Academy of Sciences, Shanghai, China).

### 2.5 RNA extraction and qRT‐PCR

Total RNA was extracted from the tissue specimens and cells using TRIzol (Invitrogen), and qRT‐PCR was performed with SYBR® Green Dye (Takara, Dalian, China) according to the manufacturer's instructions. The primer sequences are listed in Table S3.

### 2.6 Cell transfection

The lncRNA AK002107‐knockdown vector, miR‐140‐5p inhibitor, and miR‐140‐5p mimics were obtained from GenePharma (Shanghai, China). For the packaging of the construct, 293T cells were transfected with shAK002107/NC and pPACKH1 Packaging Plasmid Mix, and after 3 days, the virus particles were collected with the Lenti‐Concentin Virus Precipitation Solution according to the SBI packaging protocol. Cells were infected with the TransDux virus transduction reagent. Positively infected cells were selected with puromycin. LipoiMAX transfection reagent (Invitrogen) was used to transfect the miR‐140‐5p inhibitor according to the manufacturer's recommended protocol. Forty‐eight hours after transfection, cells were collected and used in subsequent experiments. The following shRNA sequences were used:

shAK002107‐1: 5′‐TGATACTCAGCACTAGACTAACTTCAAGAGAGTTAGTCTAGTGCTGAGTATC‐TTTTT‐3′ and shAK002107‐2: 5′‐TGCATAGCTAATCCTGTTAAAGTTCAAGAGACTTTAACAGGATTAGCTATGC‐TTTTT‐3′.

### 2.7 MTT assay

Cells were seeded into 96‐well plates at a density of 5000 cells per well. Then, 100 μL of fresh Dulbecco's modified Eagle's medium (DMEM) and 0.5 mg·mL^−1^ MTT were added to each well at 0, 24, 48, and 72 h, and the cells were incubated at 37 °C for 4 h. After replacing the medium with 100 μL of DMSO and shaking gently at room temperature for 10 min, the absorbance was measured at 570 nm to calculate the OD value.

### 2.8 Colony formation assay

For the colony formation assay, 500 cells were seeded into six‐well culture plates, gently shaken, and incubated in a 37 °C incubator with a 5% CO_2_ atmosphere for 2 weeks. Subsequently, the medium was removed, and the cells were stained with 0.1% crystal violet (Beyotime Institute of Biotechnology, Shanghai, China), after which the positive colonies (diameter > 40 μm) were imaged and counted. The differences in the colony formation abilities of different cell types were documented.

### 2.9 Transwell invasion assay

First, 5 × 10^4^ cells in serum‐free DMEM were seeded into the upper chamber of 8‐μm Transwell inserts (BD Biosciences, Franklin Lakes, NJ, USA), and DMEM containing 10% BSA was added to the lower chamber. The upper chamber was coated with Matrigel (BD Biosciences). After a 24‐h incubation at 37 °C, the cells in the upper chamber were removed, and the cells adhering to the underside of the Transwell membrane were fixed with 20% methanol and stained with 0.1% crystal violet. Then, the number of cells was counted under an inverted microscope.

### 2.10 *In vivo* tumor growth assays

Four‐ to six‐week‐old BALB/c nu/nu mice were purchased from the Center of Laboratory Animals of Beijing Vital River Laboratory Animal Technology Co., Ltd (Beijing, China). Then, 1 × 10^6^ cells were suspended in 100 μL of PBS and subcutaneously injected into the subcutis. The tumor size was monitored by measuring the volume and weight. The width and length of the neoplasm were measured with calipers weekly. The tumor volume was calculated using the following formula: length × width^2^/2. The animal experiment was approved by and performed in accordance with the Ethic Committee on the Use of Live Animals in Teaching and Research at the First Affiliated Hospital of Sun Yat‐sen University.

### 2.11 Western blot analysis

A western blot analysis was performed using standard protocols. The following primary antibodies were used: E‐cadherin (sc‐10779, Santa Cruz, CA, USA), vimentin (CST, #9116, Danvers, MA, USA), TGFBR1 (CST, #2546), and GAPDH (CST, #3136). Secondary horseradish peroxidase‐conjugated anti‐rabbit or anti‐mouse antibodies (diluted 1 : 5000; ABGENT, San Diego, CA, USA) were applied and allowed to bind the matched primary antibodies. Protein expression levels were visualized using an enhanced chemiluminescence reagent (WBKLS0500; Millipore, Billerica, MA, USA).

### 2.12 Luciferase assay

Long noncoding RNAs AK002107 and the 3′‐UTR of TGFBR1 were amplified by PCR and subcloned into the pEZX‐MT06 luciferase reporter vector (GeneCopoeia, Guangzhou, China). The potential miR‐140‐5p binding sequences were mutated using a QuikChange site‐directed mutagenesis kit (Agilent Technologies). lncRNA AK002107 fragments with the wild‐type (WT) or mutant (MUT) miR‐140‐5p binding sites were cloned to generate the pmir‐GLO‐lncRNA AK002107‐WT or pmir‐GLO‐lncRNA AK002107‐MUT plasmids, respectively. The 3′‐UTR of TGFBR1 containing the WT or MUT miR‐140‐5p binding sites was used to generate the pmir‐GLO‐TGFBR1‐WT and pmir‐GLO‐TGFBR1‐MUT plasmids, respectively. The WT (MUT) lncRNA AK002107 vector or WT (MUT) 3′‐UTR TGFBR1 vector and miR‐140‐5p or control mimics were cotransfected into 293T cells. Luciferase activity was measured using the Luc‐Pair™ Luciferase Assay Kit (GeneCopoeia, Inc.).

### 2.13 Statistical analysis

The categorical parameters were compared with the chi‐square test or Fisher's exact test and analysis of variance as appropriate. Patient survival was determined by constructing a Kaplan–Meier survival curve and analyzed using the log‐rank test. A Pearson correlation analysis was used to assess the correlations among lncRNA AK002107, miR‐140‐5p, and TGFBR1 expression. *P*‐values < 0.05 were considered statistically significant.

## 3 Results

### 3.1 High lncRNA AK002107 expression in HCC correlates with a poor prognosis

The lncRNA and mRNA expression profiles were determined using a microarray analysis to analyze the transcripts that potentially drive liver tumorigenesis. The hierarchical clustering analysis showed systematic variations in the transcript expression levels between the paired tumor and nontumor tissues from five patients with HCC (Fig. 1A). As shown in Fig. 1B, the expression levels of lncRNA AK002107 in 30 HCC tissues and corresponding noncancerous tissues were examined using real‐time PCR to validate our microarray findings. Significantly higher expression of lncRNA AK002107 was observed in the tumor tissues than in the normal tissues (*P* < 0.001). To validate this result, ISH was performed in 100 HCC tissues from the training cohort (Fig. 1C). The expression of lncRNA AK002107 was significantly upregulated in 61 HCC tissues (61%). The one hundred HCC tissues were divided into the following two groups: a high lncRNA AK002107 expression group (*n* = 61) and low lncRNA AK002107 expression group (*n* = 39). As shown in Table 1, high lncRNA AK002107 expression in HCC tissues correlated with a higher AFP level (*P* = 0.001), a larger tumor size (*P* < 0.001), macrovascular invasion (*P* < 0.001), and microvascular invasion (*P* = 0.020). A Kaplan–Meier analysis and log‐rank test were used to evaluate the effects of lncRNA AK002107 expression on overall and disease‐free survival and to evaluate the potential correlation between lncRNA AK002107 expression and patient prognosis. Patients presenting high lncRNA AK002107 expression exhibited a significantly poorer prognosis than patients with low lncRNA AK002107 expression (*P* < 0.001; Fig. 1D,E). A multivariate Cox proportional regression analysis of risk was further performed to analyze the clinicopathological characteristics of 100 patients. Based on the results of the multivariate analysis, multiple tumors, a larger tumor size (> 5 cm), and high lncRNA AK002107 expression were independent prognostic factors for overall and disease‐free survival (Table 2).

**Figure 1:** Overexpression of lncRNA AK002107 in HCC tissues. (A) Hierarchical clustering analysis of the differentially expressed lncRNAs (> 2‐fold; *P* < 0.05) between HCC samples (T, tumor) and paired nontumor samples (N, nontumor). (B) The expression of lncRNA AK002107 in thirty fresh HCC samples and adjacent noncancerous tissues was analyzed using qRT‐PCR. Results expressed as the means ± SDs. Student's *t*‐test was performed for statistical comparisons. (C) Representative images of high and low lncRNA AK002107 expression in 100 human HCC tissues analyzed using ISH (200× and 400×). Positive ISH staining for lncRNA AK002107 was blue (arrow). The length of the scale bars is 100 μm (200×) and 50 μm (400×), respectively. (D) Kaplan–Meier survival curves showing the overall survival of 100 patients with HCC classified according to their relative lncRNA AK002107 expression level; *P* < 0.001 according to the log‐rank test. (E) Kaplan–Meier survival curves showing the disease‐free survival of 100 patients with HCC classified according to their relative lncRNA AK002107 expression level; *P* < 0.001 according to the log‐rank test.

**Table 2:** Prognostic factors for DFS and OS by a multivariate Cox proportional hazards regression model. CI, confidence interval; DFS, disease‐free survival; HR, hazard ratio; OS, overall survival

Variables	DFS			OS		
	HR	95% CI	*P*	HR	95% CI	*P*
Tumor number (multiple *vs* single)	2.975	1.536‐5.761	0.001	1.993	1.011‐3.929	0.046
Size of largest tumor, cm (> 8 *vs* 5 to 8 *vs* ≤* *5)	2.486	1.743‐3.545	< 0.001	2.459	1.701‐3.555	< 0.001
lncRNA‐AK002107 expression (high *vs* low)	6.289	2.690‐14.704	< 0.001	7.994	3.609‐20.820	< 0.001

### 3.2 Downregulation of lncRNA AK002107 expression inhibits HCC cell proliferation, colony formation, and invasion *in vitro*

After detecting lncRNA AK002107 expression in six HCC cell lines, we developed BEL‐7402 and MHCC97H cell lines in which the expression of lncRNA AK002107 was stably knocked down (Fig. 2A,B). We performed MTT and colony formation assays *in vitro* and observed that compared with parallel stable cell lines containing the negative control, knockdown of lncRNA AK002107 inhibited the proliferation and colony formation capacity of the BEL‐7402 and MHCC97H cells (Fig. 2C,D). Furthermore, we performed Transwell invasion assays to determine whether lncRNA AK002107 expression modulates cell invasion. Compared with the sh‐NC group, knockdown of lncRNA AK002107 significantly attenuated the invasion of both the BEL‐7402 and MHCC97H cell lines (Fig. 2E). Thus, the downregulation of lncRNA AK002107 expression inhibits HCC cell proliferation, colony formation, and invasion.

**Figure 2:** lncRNA AK002107 promotes HCC proliferation, colony formation, and invasion *in vitro*. (A) The expression of lncRNA AK002107 in six human HCC cell lines, including MHCC97H, MHCC97L, BEL7402, SMMC7721, Hep3B, and HepG2, was upregulated compared to the normal cell line LO_2_, as determined using qRT‐PCR. *P < 0.05 and **P < 0.01. (B) The expression of lncRNA AK002107 was detected in BEL7402 and MHCC97H cells using qRT‐PCR after the transduction of lentiviruses encoding lncRNA AK002107 short hairpin RNA (shRNA)‐1, shRNA‐2, or scrambled shRNA. All qPCR results shown as data from at least two independent replicates. Statistical analyses using one‐way ANOVA with Tukey's post‐test, *P < 0.05. and **P < 0.01. (C) MTT assays were performed to assess the proliferation of the HCC cell lines BEL7402 and MHCC97H in response to transfection with lncRNA AK002107 shRNA‐1 or lncRNA AK002107 shRNA‐2 compared with the sh‐NC group. Two‐way ANOVA with multiple comparisons (Tukey's post *t*‐test) performed to measure significance, *P < 0.05. Results are from three independent experiments. (D) A colony formation assay was performed to determine the colony formation capacity of the HCC cell lines BEL7402 and MHCC97H in response to transfection with lncRNA AK002107 shRNA‐1 or lncRNA AK002107 shRNA‐2 compared with the sh‐NC group. Magnification, 200×. Error bars represent the SD of three independent experiments. Student's *t*‐test was used to statistical analyses. **P < 0.01. (E) Transwell invasion assay of BEL7402 and MHCC97H cells transfected with lncRNA AK002107 shRNA‐1 or lncRNA AK002107 shRNA‐2 compared with the sh‐NC group. The length of the scale bars is 100 μm. Error bars represent the SD of three independent experiments. Student's *t*‐test was used to statistical analyses. **P < 0.01.

### 3.3 Downregulation of lncRNA AK002107 expression inhibits HCC tumor growth *in vivo*

We established an *in vivo* xenograft model in nude mice by subcutaneously injecting BEL‐7402‐sh‐lncRNA AK002107‐1 and MHCC97H‐sh‐lncRNA AK002107‐1 cells and their corresponding controls into nude mice and monitoring tumor growth to confirm our *in vitro* findings. The xenograft tumors that developed from the BEL‐7402‐sh‐lncRNA AK002107‐1 and MHCC97H‐sh‐lncRNA AK002107‐1 cells had smaller volumes and weights and formed more slowly than the tumors that developed from the control cells (Fig. 3A–D). Based on these results, the downregulation of lncRNA AK002107‐1 expression inhibits HCC tumor growth *in vivo*. Furthermore, by performing western blot assays of the dissected tissues, lncRNA AK002107 knockdown significantly increased the levels of the epithelial marker E‐cadherin and decreased the levels of the mesenchymal marker vimentin (Fig. 3E).

**Figure 3:** Downregulation of lncRNA AK002107‐1 expression inhibits HCC tumor growth *in vivo*. (A) Representative images of tumors formed in nude mice that had been subcutaneously injected with BEL7402 or MHCC97H cells transfected with lncRNA‐AK002107 shRNA‐1 compared with the sh‐NC group. (B) The weight of tumors dissected from the shAK002107‐1 group was lower than the sh‐NC group. Data are shown as means ± SD, and Student's *t*‐test was used to calculate significance, *P < 0 .05. (C) The tumor volumes were significantly reduced at 1, 2, 3, and 4 weeks following the injection of shAK002107‐1‐expressing tumor cells compared with the sh‐NC group. Data are shown as means ± SD, and Student's *t*‐test was used to calculate significance,*P < 0.05. (D) Representative ISH image showing lncRNA AK002107 shRNA‐1 expression in xenograft tumors from nude mice injected subcutaneously with BEL7402 or MHCC97H cells transfected with lncRNA AK002107 shRNA‐1 construct compared with the sh‐NC group. The length of the scale bars is 50 μm. (E) Levels of the E‐cadherin and vimentin proteins in xenograft tissues were determined using western blotting.

### 3.4 MiR‐140‐5p is a direct target of lncRNA AK002107 in HCC

Interactions between lncRNAs and microRNAs (miRNAs), which are pivotal classes of noncoding RNAs in eukaryotes, provide an additional layer of control of gene expression (Tay *et al*., 2014). A cohort of nine miRNAs (miR‐27a‐3p, miR‐27b‐3p, miR‐128‐3p, miR‐140‐5p, miR‐203a‐5p, miR‐216a‐3p, miR‐219b‐5p, miR‐331‐3p, and miR‐412‐3p) that potentially interact with lncRNA AK002107 was predicted using the STARBASE 2.0 and miRanda databases (http://starbase.sysu.edu.cn/ and http://www.microrna.org/, respectively). Among these miRNA candidates, lncRNA AK002107 directly binds to miR‐140‐5p, and the expression of miR‐140‐5p was reduced to the greatest extent in the miRNA profiling assay; thus, we selected miR‐140‐5p for further analysis. The site in miR‐140‐5p to which lncRNA AK002107 binds was identified (Fig. 4A). Furthermore, the luciferase reporter assay revealed that miR‐140‐5p significantly decreased the luciferase activity of the lncRNA‐AK002107‐WT vector compared with the lncRNA‐AK002107‐MUT vector (*P* < 0.05, Fig. 4B). Then, miR‐140‐5p expression in HCC cells was determined using real‐time PCR assays (Fig. 4C). BEL‐7402 and MHCC97H cell lines with stably silenced miR‐140‐5p expression were generated. We further investigated the regulatory relationship between lncRNA AK002107 and miR‐140‐5p. Knockdown of lncRNA AK002107 significantly increased miR‐140‐5p expression in the BEL‐7402 and MHCC97H cells (Fig. 4D), suggesting that lncRNA AK002107 inhibits miR‐140‐5p expression.

**Figure 4:** MiR‐140‐5p is a target of lncRNA AK002107. (A) Bioinformatics analysis identified the putative binding sites for lncRNA AK002107 in the miR‐140‐5p sequence. (B) Luciferase activity was determined in 293T cells cotransfected with miRNAs (control mimics or miR‐140‐5p mimics) and a reporter vector containing lncRNA AK002107 segments (WT or MUT) that bind to miR‐140‐5p. *P < 0.05. (C) The expression of miR‐140‐5p in six human HCC cell lines, including MHCC97H, MHCC97L, BEL7402, SMMC7721, Hep3B, and HepG2, was downregulated compared to the normal cell line LO_2_, as determined using qRT‐PCR. *P < 0.05 and **P < 0.01. (D) The expression of miR‐140‐5p was detected in BEL7402 and MHCC97H cells using qRT‐PCR after the transduction of lentiviruses encoding lncRNA AK002107 short hairpin RNA (shRNA)‐1, shRNA‐2, or scrambled shRNA. All qPCR results shown as data from at least two independent replicates. Statistical analyses using one‐way ANOVA with Tukey's post‐test, *P < 0.05 and **P < 0.01.

### 3.5 lncRNA AK002107 functions in HCC cell proliferation and invasion by negatively regulating miR‐140‐5p expression

We further examined whether lncRNA AK002107 functions through miR‐140‐5p. Initially, compared to the control group, knockdown of lncRNA AK002107 inhibited the proliferation and invasion of the BEL‐7402 and MHCC97H cells, and miR‐140‐5p inhibition significantly increased the proliferation (Fig. 5A) and invasion (Fig. 5B) of the BEL‐7402 and MHCC97H cells. However, this effect was reversed by the simultaneous cotransfection of sh‐lncRNA‐AK002107 and the miR‐140‐5p inhibitor (Fig. 5A,B). Thus, lncRNA AK002107 functions as an oncogene in HCC cells by regulating miR‐140‐5p expression.

**Figure 5:** lncRNA AK002107 plays a role in HCC cell proliferation and invasion by negatively regulating miR‐140‐5p expression. (A) MTT assays were performed to assess the proliferation of the HCC cell lines BEL7402 and MHCC97H in response to the transfection of lncRNA AK002107 shRNA‐1, lncRNA AK002107 shRNA‐2, or miR‐140‐5p inhibitors or cotransfection of sh‐lncRNA‐AK002107‐1 or sh‐lncRNA‐AK002107‐2 with miR‐140‐5p inhibitors compared with the sh‐NC group. Two‐way ANOVA with multiple comparisons (Tukey's post *t*‐test) performed to measure significance, *P < 0.05. Results are from three independent experiments. (B) Transwell invasion assay of BEL7402 and MHCC97H cells transfected with lncRNA AK002107 shRNA‐1, lncRNA AK002107 shRNA‐2, or miR‐140‐5p inhibitor or cotransfection of sh‐lncRNA‐AK002107‐1 or sh‐lncRNA‐AK002107‐2 with miR‐140‐5p inhibitors compared with the sh‐NC group. The length of the scale bars is 100 μm. Error bars represent the SD of three independent experiments. Student's *t*‐test was used to statistical analyses. *P < 0.05 and **P < 0.01.

### 3.6 lncRNA AK002107 modulates the expression of the miR‐140‐5p target TGFBR1 and induces epithelial–mesenchymal transition

Using targetscan software (http://www.targetscan.org/vert_72/), we found that miR‐140‐5p directly binds TGFBR1 (Fig. 6A). The miR‐140‐5p mimics reduced the luciferase activity of the WT TGFBR1 3′‐UTR in the luciferase reporter assay but had no effect on the MUT one (Fig. 6B). Next, we examined whether lncRNA AK002107 modulates the expression of TGFBR1 by targeting miR‐140‐5p in HCC cells and subsequently inducing EMT. Compared to the control group, levels of the TGFBR1 mRNA and protein were decreased in lncRNA AK002107‐silenced BEL‐7402 and MHCC97H cells and were increased in cells transfected with the miR‐140‐5p inhibitors. In the group cotransfected with the miR‐140‐5p inhibitor and lncRNA AK002107 knockdown plasmid, the modulatory effects of lncRNA AK002107 on TGFBR1 expression were diminished (Fig. 6C). Furthermore, using western blot assays, knockdown of lncRNA AK002107 significantly increased the levels of the epithelial marker E‐cadherin and decreased levels of the mesenchymal marker vimentin, while the miR‐140‐5p inhibitor significantly decreased E‐cadherin levels and increased vimentin levels. However, the miR‐140‐5p inhibitor significantly abolished the increase in E‐cadherin levels and decrease in vimentin levels induced by the knockdown of lncRNA AK002107 (Fig. 6D). Based on these results, lncRNA AK002107 negatively modulates miR‐140‐5p expression and targets TGFBR1 to induce EMT in HCC.

**Figure 6:** lncRNA AK002107 modulates the expression of miR‐140‐5p, targets TGFBR1, and induces EMT. (A) The putative binding sites between TGFBR1 and miR‐140‐5p. (B) Luciferase activity was determined in 293T cells cotransfected with miRNAs (control mimics or miR‐140‐5p mimics) and a reporter vector containing TGFBR1 3′‐UTR segments (WT or MUT) that bind to miR‐140‐5p. Error bars represent the SD of three independent experiments. Student's *t*‐test was used to statistical analyses. *P < 0.05 (C) TGFBR1 expression was detected in BEL7402 and MHCC97H cells using qRT‐PCR after the transduction of lentiviruses encoding lncRNA AK002107 short hairpin RNA (shRNA)‐1, shRNA‐2, or miR‐140‐5p inhibitor, cotransfection of the miR‐140‐5p inhibitor and sh‐lncRNA‐AK002107‐1, and cotransfection of the miR‐140‐5p inhibitor and sh‐lncRNA‐AK002107‐2 or scrambled shRNA. Error bars represent the SD of three independent experiments. Student's *t*‐test was used to statistical analyses. *P < 0.05 and **P < 0.01. (D) Levels of the E‐cadherin, vimentin, and TGFBR1 proteins were determined in BEL7402 and MHCC97H cells transfected with lentiviruses encoding sh‐lncRNA‐AK002107‐1, sh‐lncRNA‐AK002107‐2, or miR‐140‐5p inhibitor, cotransfection of the miR‐140‐5p inhibitor and sh‐lncRNA‐AK002107‐1, or cotransfection of the miR‐140‐5p inhibitor and sh‐lncRNA‐AK002107‐2 or scrambled shRNA using western blot assays.

### 3.7 Correlations between the expression of lncRNA AK002107 and miR‐140‐5p and TGFBR1 levels in human HCC tissues

We analyzed miR‐140‐5p and TGFBR1 expression in 30 HCC tissues and corresponding noncancerous tissues using real‐time PCR. The expression of miR‐140‐5p was significantly decreased in the HCC tissues compared with the corresponding tumor‐adjacent nontumor tissues (Fig. 7A). Furthermore, an inverse correlation was identified between lncRNA AK002107 and miR‐140‐5p expression levels (*r* = −0.596, *P* = 0.0005; Fig. 7B). Based on the real‐time PCR data, TGFBR1 expression was significantly increased in the 30 HCC tissues compared with the corresponding tumor‐adjacent nontumor tissues (Fig. 7C). Furthermore, a positive correlation was identified between lncRNA AK002107 and TGFBR1 expression levels (*r* = 0.516; *P* = 0.0035; Fig. 7D). Therefore, lncRNA AK002107 plays a functional role in inducing EMT by inhibiting miR‐140‐5p expression and subsequently upregulating TGFBR1 expression in HCC (Fig. 7E).

**Figure 7:** Expression of miR‐140‐5p and TGFBR1 and the correlations between lncRNA AK002107 and miR‐140‐5p and TGFBR1 expression in HCC tissues. (A) The expression of miR‐140‐5p was analyzed in thirty fresh HCC samples and adjacent noncancerous tissues using qRT‐PCR. Results expressed as the means ± SDs. Student's *t*‐test was performed for statistical comparisons. *P* < 0.0001, (B) Correlations between the expression of lncRNA AK002107 and miR‐140‐5p were analyzed using Spearman's rank correlation analysis. (C) TGFBR1 expression in thirty fresh HCC samples and adjacent noncancerous tissues was analyzed using qRT‐PCR. Results expressed as the means ± SDs. Student's *t*‐test was performed for statistical comparisons. *P* = 0.006. (D) Correlations between the expression of lncRNA AK002107 and TGFBR1 were analyzed using Spearman's rank correlation analysis. (E) Schematic of the lncRNA AK002107/miR‐140‐5p/TGFBR1/EMT regulatory network in HCC.

## 4 Discussion

The key finding of this study is that the expression of lncRNA AK002107 is upregulated in HCC tissues compared to corresponding noncancerous tissues. High lncRNA AK002107 expression in HCC correlated with a poorer prognosis. The downregulation of lncRNA AK002107 expression significantly inhibited HCC cellular proliferation, colony formation, and invasion both *in vitro* and *in vivo*. lncRNA AK002107 increased the level of TGFBR1 and then induced EMT in HCC by inhibiting miR‐140‐5p expression. Thus, based on our results, lncRNA AK002107 functions as an oncogene in HCC and should be considered a potential prognostic indicator.

According to emerging evidence, lncRNAs function as key regulators of carcinogenesis and cancer progression (Hu *et al*., 2017). However, only a few lncRNAs have been confirmed to perform various functions in HCC (Shi *et al*., 2016). In the present study, we first identified that a novel lncRNA (AK002107) functioned as an oncogene in HCC. The expression of lncRNA AK002107 was frequently upregulated in clinical HCC tissues and cell lines. The expression of lncRNA AK002107 correlated with aggressive clinicopathological characteristics and was an independent risk factor for disease‐free survival and overall survival. Patients with elevated lncRNA AK002107 expression exhibited significantly shorter overall survival and higher recurrence rates than patients with low AK002107 expression. Next, we investigated whether lncRNA AK002107 functions in HCC cells. This lncRNA was found to promote HCC proliferation, colony formation, and invasion *in vitro* and *in vivo*. Therefore, aberrant expression of lncRNA AK002107 accelerates HCC progression in both human HCC tissues and cells. These data support our conclusion that lncRNA AK002107 possesses oncogenic activity.

An understanding of RNA crosstalk provides significant insights into gene regulatory networks and has implications in cancer (Guil and Esteller, 2015). Notably, lncRNAs and miRNAs interact with and coregulate each other through multiple mechanisms (Tay *et al*., 2014) by acting as competing endogenous RNAs or natural miRNA sponges that compete for binding to shared miRNAs. The interactions between lncRNAs and miRNAs have been recently studied and aroused interest. We aimed to reveal the regulatory mechanism of lncRNA AK002107 in HCC; here, we present strong evidence that lncRNA AK002107 promotes HCC progression by targeting miR‐140‐5p. lncRNA AK002107 competitively binds miR‐140‐5p to suppress its effects. Knockdown of lncRNA AK002107 significantly increased miR‐140‐5p expression and inhibited HCC progression, which was counteracted by miR‐140‐5p silencing. Based on these results, lncRNA AK002107 functions as an oncogene by regulating miR‐140‐5p expression. As shown in previous studies, miR‐140‐5p acts as a tumor suppressor in many cancers, such as lung cancer (Polley *et al*., 2016), gastric cancer (Cui *et al*., 2017), osteosarcoma (Wei *et al*., 2016), and ovarian cancer (Lan *et al*., 2015), consistent with our finding that miR‐140‐5p exerts an inhibitory effect on HCC in the current study. In clinical HCC tissues, the expression of lncRNA AK002107 and the expression of miR‐140‐5p were inversely correlated, further verifying that miR‐140‐5p is a direct target of lncRNA AK002107 in HCC.

In this study, lncRNA AK002107 modulated the expression of the miR‐140‐5p target TGFBR1 to induce EMT and promote HCC progression. According to (Yang *et al*. (2013) miR‐140‐5p suppresses the growth and metastasis of HCC by inhibiting TGFBR1 and FGF9 expression, and TGFBR1 has been identified as a promoter of cancer cell growth by inducing EMT (Han *et al*., 2005; Thien *et al*., 2015). We monitored the protein and RNA levels of TGFBR1 following AK002107 knockdown and miR‐140‐5p inhibition to confirm that lncRNA AK002107 and miR‐140‐5p coordinately regulate the TGFBR1/EMT pathway in HCC cell lines. Knockdown of lncRNA AK002107 decreased TGFBR1 and vimentin levels and increased E‐cadherin levels, which inhibited EMT. However, the cotransfection of cells with a miR‐140‐5p inhibitor and shRNA targeting lncRNA AK002107 reversed the expression patterns of these EMT‐related proteins. In HCC cell lines, lncRNA AK002107 was found to affect HCC cell proliferation, colony formation, and invasion through a miR‐140‐5p‐dependent TGFBR1/EMT pathway. Moreover, in clinical HCC tissues, miR‐140‐5p expression was downregulated, while the expression of lncRNA AK002107 and TGFBR1 was upregulated. lncRNA AK002107 expression inversely correlated with miR‐140‐5p expression and positively correlated with TGFBR1 expression, further confirming that this lncRNA targets miR‐140‐5p to suppress its expression, which subsequently upregulates TGFBR1 and induces EMT to promote HCC progression.

## 5 Conclusion

In summary, novel lncRNA AK002107 is significantly upregulated in HCC, competitively inhibits miR‐140‐5p, and subsequently upregulates the expression of its target gene, TGFBR1, to promote the proliferation, colony formation, and invasion of HCC. The lncRNA AK002107/miR‐140‐5p/TGFBR1/EMT regulatory network may be vital for tumorigenesis in HCC and may be a valuable target for the development of novel diagnostic and treatment methods for HCC.

## Conflict of interest

The authors declare no conflict of interest.

## Author contributions

YHT, GLH, SZH, YG, ZWP, and SJF were the main authors of the manuscript. They were involved in the conception, design, and coordination of the study; data analysis; interpretation of results; and drafting the manuscript. YHT, GLH, and SZH were in charge of all experimental procedures. KBZ, HL, and LC participated in the experimental procedures and revised critically the content of the manuscript. All authors contributed to the interpretation of data and critically revised the manuscript. All authors read and approved the final manuscript.

## Supporting information


**Table S1**. Basic characteristics of the five patients with HCC included in the lncRNA/mRNA analysis.

**Table S2**. Clinicopathological characteristics of 30 patients with HCC.

**Table S3**. Primer sets used for qRT‐PCR.
